The article "Recognition Method of Wushu Human Complex Movement Based on Bone Point Feature" was published in 2022. Journal: Comput Math Methods Med.

# Recognition Method of Wushu Human Complex Movement Based on Bone Point Feature

**DOI:** 10.1155/2022/2287991

**Published:** 2022-04-21

**Authors:** Anping Li, Ruijie Zhang, Lingrong Tao

**Affiliations:** ^1^Department of Physical Education and Research, Yang-En University, Quanzhou 362014, China; ^2^Department of Physical Education, Tangshan Normal University, Tangshan 063000, China; ^3^Graduate School of Jeonju University, Jeonju 54800, Republic of Korea; ^4^Physical Education Institute, Jimei University, Xiamen 361021, China

## Abstract

The existing recognition methods of complex human movements in Wushu have the problem of imperfect kinetic energy model, which leads to low recognition accuracy. A complex human motion recognition method based on bone point features is designed. Identify martial arts movement posture, combine the upward movement of human center of gravity trajectory, establish the kinetic energy model of joints according to the positioning results of extremity points, set the threshold of local spatial differences of human bones with the central node of hip joint as the center point, avoid overcalculation, and optimize the complex motion identification process by combining the characteristics of bone points. *Experimental Results*. The correct rate of different types of actions identified by this method is 90.1% and 92.7%, and the identification time is 1.2 s and 1.41 s, which shows that this method can identify actions quickly and effectively by combining the feature information of bone points.

## 1. Introduction

Human complex motion recognition is developed on the basis of human motion recognition. Human movement is a highly complex nonrigid body movement, which presents complex characteristics during human movement. As a result of the different body shape, movement habits, and different people do, the same movement will have obvious differences, which undoubtedly increases the technical difficulty for human movement recognition. In order to describe the human movement more truly and to facilitate calculation, most of the present use of human body model to represent, that is, human skeleton model. Humans can sense and capture movement information through the eyes, ears, and other organs, then analyze the movement information through the brain, and judge the movement according to their own experience. The human action recognition algorithm imitates the process of human action recognition, automatically detects and analyzes human actions from the action sequence data collected by various sensors, and inferences their semantic information. In daily life, it is very simple to recognize human movements by the naked eye. However, it is a very complicated and challenging task to realize automatic classification of human movements by computer vision system. Among them, there are many problems to be solved, such as the capture of human action information, the learning of training samples, the recognition of small changes of similar action patterns in time and space, and the acquisition of human behavior intentions. In the traditional action recognition, human eyes are used to watch the action sequence to recognize the action, which has low efficiency and large error and cannot meet the processing requirements and efficiency of today's action sequence recognition. At present, human motion recognition technology is not mature enough, and there is still a long way to go. Some scholars have proposed some action recognition methods, such as Sucipto et al. [1], which put forward the advantage of multilayer operation of neural network to realize action recognition. Tirtasari et al. [2] proposed to design a motion recognition method by using the iterative calculation theory of deep learning.

In some traditional martial arts, the movement range is large and the movement posture is complex, such as Tai Ji Chuan and other martial arts sports, which include routine movements. The martial arts posture can be obtained through the decomposition of movement recognition, so as to evaluate the standardization of movements and correct the wrong movements, so that practitioners can reach the best standard. The main difficulties of this research are as follows: human body structure and motion. The human body is a complex organism composed of a series of bone joints, and its motion is composed of different postures driven by related bones. Experts generally need about 60 joint parameters of the human body model to achieve accurate estimation of human motion, but the calculation of optimal parameter estimation in the parameter space of more than 60 dimensions is very complicated and requires a lot of time. Therefore, the subject of Wushu human complex movement recognition needs to be further discussed. In this paper, a recognition method of complex movements of Wushu human body based on the characteristics of bone points is proposed. Taking the extremities and joints as nodes, a human movement model is constructed. Considering the complexity of movements in Wushu, the threshold constraint on the posture space of human movement is increased, which greatly reduces the amount of calculation, thus realizing the recognition of Wushu movements.

## 2. Recognition Method of Wushu Human Complex Movement Based on Bone Point Feature

### 2.1. Identifying Martial Arts Gestures

Take the aerial movement in martial arts as an example. The aerial leg combination requires swinging the right leg higher than the shoulder and striking the left hand loudly [3–5], as shown in Figure 1.

So kick the right leg as high as possible, and speed up the swing to hit the left hand. In this case, a high kick on the right leg requires flexibility. Otherwise, not only will the right leg not be close to the body but the left leg left behind will bend forward as the kick on the right leg is high. In addition, at the beginning of the air, the right leg should be swung from the right down to the left. At the beginning of starting, the distance between the right leg and the longitudinal axis is the largest, and the impact on the rotational angular acceleration is also the largest. Therefore, the duration of this period should be minimized as far as possible. This puts a high demand on the explosive strength of the muscles responsible for horizontal flexion and adduction of the hip joint. These muscles have good explosive force, so they can quickly complete the swing action of the right leg and reduce the duration of the moment of inertia increase, which is conducive to the increase of rotational angular acceleration. Compared with routine movements, the biomechanics research of Sanda is more explicit and direct in the discussion of the attack and technique of movements. For example, it is pointed out that the final effect of the end leg is determined by “the hitting power and speed at the end of the link” when using the change of toe speed to evaluate the effect of the side rising leg in Sanda. According to the above theory, it can be seen that the movement of the closed leg in the air is contradictory to the important purpose of the cyclonic foot 720° catch step, that is, to complete the rotation of 720° around the longitudinal axis of the human body. The inside leg movement increases the difficulty of rotation, and if you do not pay attention to the posture of the leg, it will easily affect the quality of the movement. Therefore, the air leg movement is one of the difficulties of the whole movement. In order to complete the in-air leg movement and minimize the impact on the air rotation, it is necessary to have a good flexibility of the right leg and even the left leg. During the in-air leg movement, the legs should be kept as straight as possible to reduce the moment of inertia. The main generating muscles in the buffering stage are shown in Figure 2.

As can be seen from Figure 1, the main generating muscles in the buffering stage are vastus lateralis, rectus femoris, vastus medialis, tibialis anterior, gastrocnemius, and gluteus maximus. After comparing the strength of side rui leg of the first class Sanda athlete with that of the master class, the importance of side rui leg strength is found. The test results are influenced by such factors as whether to hit directly with empty hands, wearing gloves of different materials, hand binding bandages of different textures, and the thickness of cushion on the surface of force measuring instrument. At the same time, it is necessary to make the right leg horizontal flexion and adduction of the muscle with good explosive force, so that the right leg as soon as possible completes the body swing action. As is known to all, boxing, like martial arts, can directly hit the head and torso of the opponent, and the ability of the head to withstand continuous blows directly affects the result of the match [6, 7]. The data showed that, under selected conditions of 22 boxers, each fighter struck a Kistler bench containing an air cushion 10 times, using an electrooptical system to measure the rate of the strike. After the ring, the links of the human body, and downward movement, the track of the center of gravity is also downward, so the movement of the human body links with the track of the center of gravity. At the same time, because of the human body after been smacked his right leg and left hand part requirement for fast lap to reduce the rotation radius, thus make human body center of gravity relative to the position of the human body the hem of the link fast down, down track down faster than the speed of heart, so cause the human body after been smacked hem links human heads up on the top of the phenomenon, this is called “secondary” suspension, some research. The second aerial can make the aerial movement stretch and elegant feeling, which is beneficial to improve the appreciation of the movement and the evaluation of the quality of the movement. It can be seen from the above that when the kicking point in the air is selected at the highest point of the center of gravity motion track, the link's motion can be matched with the center of gravity motion track to achieve the optimal motion effect [8, 9]. The results showed that the increase in force was related to the thickness of the bandage, and that bandages containing lead plaster had a greater impact on force than thin bandages. Based on the above description, complete the steps of identifying martial arts gestures.

### 2.2. Building the Kinetic Energy Model of Key Nodes

People's different actions are not only shown in the difference of position information but also in the energy characteristics of the sequence of junctions. This paper proposes a new skeletal expression for behavior recognition. Inspired by the law of kinetic energy and gravitation, this paper finds that kinetic energy and potential energy can effectively represent the change of human energy. According to the characteristics of human skeleton joints, joints are divided into three categories: skeleton end points, trunk end points, and inflection points of limbs. The end points of the skeleton include the extremities and head with five points in total, the neck joint and hip joint are the end points of the trunk, and the inflection points of the limbs include the elbow joint and knee joint with four points in total. Different methods are used to locate the three key nodes. This energy change provides a more meaningful feature description than a single bone feature, so in this paper, energy information and bone joint information are combined as a new feature, namely, hybrid joint feature. In the process of action recognition, human behavior states can be divided into two types: static and motion. When a person changes from a static state to a moving state, the location information of multiple nodes will change. At this time, all these nodes have moving speed. The 8-neighborhood method is used to calculate the 8-neighborhood pixel values of skeleton pixels and locate joint endpoints. According to the result of locating the extremities, an improved chain code traversal structure was used to traverse the human skeleton and locate the extremities. In order to calculate the kinetic energy of human skeleton joints, the three-dimensional coordinates of human skeleton joints should be obtained first, and then, the kinetic energy of human skeleton joints of each frame should be calculated according to the changes of coordinate information of two adjacent frames. The calculation formula is as follows:

(1) $$\begin{array}{c} G=\left\{\begin{array}{c} {{wr}_{\beta }}^{2}\\ \frac{\beta {\left|r-w\right|}^{2}}{\Delta r^{2}} \end{array}\right.. \end{array}$$

In formula (1), *w* represents kinetic energy parameter, *r* represents the time interval between two adjacent frames, and *β* represents kinetic energy of the *β* node. Under different behaviors, the kinetic energy of the joints of human body also shows different change rules. For example, the kinetic energy of the joints of human body changes greatly and changes quickly when people kick, while the kinetic energy of the joints of human body changes relatively gently, and the change frequency is low when people jog. Therefore, it can be seen intuitively that the kinetic energy of joints is an important feature of human behavior recognition [10–12]. According to the length proportion of each part of the anatomy of the human body and the result of locating the end of the trunk, the joint proportion is used to locate the inflection point of the limbs. Under the condition that the velocity has been converted into kinetic energy as an important characteristic information, the direction change vector of each joint is calculated according to the coordinates of three-dimensional joints, and the calculation formula is as follows:

(2) $$\begin{array}{c} \gamma =T_{\beta ,\beta -1}-e. \end{array}$$

In formula (2), *T* represents the spatial position of the gateway node, *e* represents the three-dimensional coordinates of the gateway node in *T* frames, and *β* has the same meaning as formula (1). The main movement of human body is limb movement. The main body is basically vertical and has a large slope relative to the horizontal direction. According to the data analysis, the burrs are generally located on both sides of the main body, and there is a certain angle relative to the main body, but the slope relative to the horizontal direction is smaller than the main body. Human behaviors are not only related to human's current location information but also related to past location information [13, 14]. For example, when describing the motion state of the legs, the motion speed and rotation direction of the legs are usually described. Similarly, in behavior recognition, each node should not only consider the speed of each node in a frame but also consider the movement direction of the node [15, 16]. According to the body structure of human body, the head node is selected as the reference point of zero potential energy in this paper. The head node is better and easier to calculate as the reference point of zero potential energy. The human attitude potential energy is defined as follows:

(3) $$\begin{array}{c} L=Q\frac{\left(\left|s-\delta_{r}\right|\right)}{2}. \end{array}$$

In formula (3), *Q* represents potential energy parameter, with a value of 9.6; *s* represents the position of the *s* junction; *δ* represents the position of the reference point of zero potential energy at the head junction; *r* has the same meaning as formula (1). In different behavior states, the speed of movement of the node is different at different moments, and the direction of change may also be different. Based on this feature, slope constraint is introduced in this paper. When the branch length is greater than the burr threshold, the slope of the branch relative to the horizontal direction is calculated, and only when the branch slope is less than the slope, threshold is judged as burr. The slope constraint can avoid misjudgment of the shorter trunk, accurately remove burrs, and preserve the intact skeleton body. Since the coordinate of the joint is relative to that of the camera, the coordinate value of the joint of the same person and the same action will differ greatly due to the different position of the camera. Considering that the human posture is mainly determined by the relative position of each part of the human body, if a relatively stable motion point is taken on the human body as a reference point, the relative coordinate of each node is calculated to eliminate the influence caused by the different relative position of the human and the camera. Based on this, the steps of constructing the kinetic energy model of the joint are completed.

### 2.3. Setting the Threshold of Local Space Difference of Human Skeleton

The information of human skeleton not only reflects the local shape of human body but also describes the topological information of human body structure. Due to the complex structure of the human skeleton model, there are more than 200 bones in total, and each bone node has different degrees of freedom, so it is difficult to model the movement using the actual human skeleton model. In the feature vector that expresses human posture based on skeleton data extraction, the attribute characteristic value of the same dimension presents multiple continuous curves for different types of actions with the passage of action execution time. Based on the physical characteristics of movement, we regard the movement of human body as a movement of bone points, each of which is independent and interconnected [17–19]. When calculating the angle, considering that most of the movement is the movement of the limbs, the changes in these parts can provide more information for describing the movement of the human body. Eight sets of nodes are specified, and the corresponding angles are calculated for each set as shown in Table 1.

As can be seen from Table 1, in order to overcome the change of spatial information of key nodes caused by the change of position of human body relative to the camera in the process of movement, it is necessary to adjust the information of human skeleton and determine the new coordinate system. However, the curves may be nearly identical at some times and very different at others. This is because there are similar parts at different time stages in the execution process of different types of actions, and these features make very little or redundant contributions to the subsequent action recognition. Therefore, we should not only obtain the spatial motion information between bone points but also pay attention to the spatial geometry information. Due to the topological structure of human skeleton, it is necessary to fully consider the motion change information of the node. The method proposed in this chapter takes the hip central node as the center origin and obtains the calculation formula of the initial spatial position characteristics as follows:

(4) $$\begin{array}{c} D=\frac{1}{W_{\varepsilon }-W_{O}}\left(\varepsilon =1,2,3,\cdots ,N\right). \end{array}$$

In formula (4), *W*_*ε*_ represents other bone nodes except the hip center point, *W*_*O*_ represents the hip center point, and *N* represents constant. In this method, the coordinates of other points are subtracted from the origin, respectively; that is, the coordinates of the three coordinate axes of the corresponding point are subtracted from the coordinates of the central point of the hip. For example, on the *x*-axis,

(5) $$\begin{array}{c} \Delta x_{\varepsilon }^{N}=x_{\varepsilon }^{N}-x_{O}^{N}. \end{array}$$

In formula (5), *x* represents the link point of the feature vector of the image. In the original high-dimensional feature space, the characteristic values of a given action sample in different time dimensions have temporal correlation. However, due to the difference in human height, people with different height have different skeleton sizes. Therefore, the data we get may differ greatly and lead to false identification. In other words, the taller a person is, the longer his bone segments are. Therefore, when extracting information from human skeleton, we must take into account the size of the skeleton and establish a normalized mechanism:

(6) $$\begin{array}{c} \bar{\lambda }=\frac{\lambda }{U}. \end{array}$$

In formula (6), *λ* represents the absolute length from the head to the spine, and *U* represents the spatial location features obtained. That is, with the execution of the action, the same eigenvalue will form a continuous state curve with the passage of time. The joint is the joint of two or more bone segments, and the bone angle formed by these bone segments indirectly reflects the movement changes between bone segments. Therefore, the angle at the bone joint is also an important feature of human movement. The position of each part of the human body in space will change differently, but some parts will not change relatively [20]. For different types of actions, the characteristic amplitudes and variation trends of some time periods are quite different, while some time periods are basically the same or similar, which has great redundancy for the subsequent discrimination and analysis of actions and affects the efficiency of decision-making. In order to describe the position characteristics of bone points during human movement, the motion features were extracted by using the spatial position information of joints. When the body completes the movement, the relative position of the nodes will change accordingly. For example, in the waving movement, the wrist joint is below the shoulder joint at the beginning. Through principal component analysis, redundancy is removed, and only feature data of dimensions with large differences are retained as the basis of decision discrimination. The principal components extracted from one kind of action samples are weighted and summed by the attribute values of the original feature vectors in different time dimensions. It can be proved that the interclass variances of action samples of different types are large in the principal component dimensions that are arranged according to the size of the feature values. However, in the process of arm lifting, the relative positions of the two nodes change significantly. By concretizing this change, that is, obtaining the characteristics of position change to describe the movement, it is of great significance to analyze the motion state. Based on the above description, the steps of setting the threshold of local spatial difference of human skeleton are completed.

### 2.4. Bone Point Features Optimizing Complex Motion Recognition Processes

From the perspective of bone point features, Kinect can extract 20~25 bone joint features of the human body, and different human movements will also involve changes in different joint angles [21–23]. Because the movement of human body is caused by the mutual drive of each skeleton, the movement of human body can be regarded as a rigid complex movement to a certain extent. Bone angle features are closely related to this property. We applaud and drink water; these two movements, in fact, mainly involve the angle between the wrist and arm, as well as the elbow angle between the size of the arm, and arm and shoulder angle, and Wushu also involves the lower body of the foot joint angle change. Complex motion features refer to the relevant parameters extracted from human motion sequences that can correctly describe human motion states. Human body image color, texture, tracking to information, such as the kinematics characteristics can be as a human motion characteristic parameters of common characteristic parameters include the speed of the human body joint, polar radius distance, angles and coordinates of joint Angle as a further advantage of features are: goals are translations or rotations, relative joint coordinates, not involved in any joint Angle change. Generally speaking, motion recognition is classified according to different categories of human motion sequence. Human motion recognition process is shown in Figure 3.

As can be seen from Figure 3, feature extraction refers to the extraction of relevant action information from human action sequence, and feature representation refers to the organic combination of complex action feature information in a special way. Action classification refers to the classification of human action sequences tested into corresponding action classes [24]. Here, we regard the bone model as composed of many bone segments. Adjacent bone segments are connected by bone points, and the degrees of freedom at different bone points are relatively different. For example, the elbow bone has a higher degree of freedom, while the knee bone has a lower degree of freedom than the elbow bone. Here, bone angle and bone vector are defined first. In this chapter, 14 angles in the human skeleton are taken, and each angle is calculated by two bone vectors. As the recognition of complex human actions depends on the characteristic parameter information of these actions, relevant characteristic parameters should be selected or constructed according to the specific properties of the object to be identified [25, 26]. In complex motion feature extraction, motion feature extraction can be divided into nonmodel and model-based methods based on whether human body model is needed or not. Model-based method is formed on the basis of nonmodel method. In order to contain as much information as possible, many human epigenetic features are often selected because of the difference in the action characteristics reflected by each epigenetic feature. Since the change of bone angle of wrist and foot is of little significance for motion recognition, and considering the amount of calculation, the included angle feature of these four bones (left and right wrist and left and right foot) is not used here. Since the angle between bones is the angle between two adjacent bones, we need to use the vector of partial bone segments in the skeleton. Generally speaking, the more information the selected complex motion features contains, the more accurate the human motion described will be, and the higher the recognition rate of complex motion will be. Motion is a time-varying signal, and motion recognition is a classification problem of time-varying signals. Complex action recognition can be described as matching test sequence with sample sequence of known action type to get the action type of test sequence, and it can deal with slight feature changes in time scale and space in similar action categories. Based on this, the steps of optimizing the complex action recognition process are completed.

## 3. Application Testing

### 3.1. Selecting Data Set

The action recognition data set used in this project comes from the real-time collection of data of people with different action types and different body types and forms CSV files after normalization. There are a total of 33 columns, the first 28 are the two-dimensional coordinate information of 16 key points, and the last one is the action category label. Since it is tedious to write by neural network program in C#, we adopt the feedforward program that only writes neural network in C#, and the training program of neural network is written in python environment. In order to make the data diversified, the data set includes the data of people of different heights and sizes. There are 2763 items in all data sets, including 540 items for standing, 525 items for kicking, 553 items for waving, 555 items for starting, and 590 items for preparing. This topic is verified in the Intel^®^ Core™ I7-3470 CPU@3.20GHz, 8GB memory environment. The operating system is 64-bit Windows 10, and the experimental tools are the Python editor Pycharm, the code editor Sublime Text, and the enhanced command line tool Cmder in Python. We set up a 3-layer neural network with 13 neurons in the first hidden layer, 14 neurons in the second hidden layer, and 10 neurons in the output layer. The activation function used by the neural network is sigmoID function. The result recognition effect is shown in Figure 4.

### 3.2. Test Result

In order to verify the effectiveness of the martial arts human body complex action recognition method in this paper, experimental tests are carried out to test the recognition accuracy of the three recognition methods under different data sets. The three data sets are msraction-3d data set and florence3d action data set. Select the martial arts human body complex action recognition method based on neural network (Literature [8] method) and the martial arts human body complex action recognition method based on deep learning (Literature [9] method), and compare it with the martial arts human body complex action recognition method in this paper. The test results are shown in Figures 5 and 6.

As shown in Figure 5, the average accuracy rate of the martial arts human movement recognition method in this paper is 90.1%, and the average accuracy rates of the other two recognition methods are 78.2% and 76.5%, respectively. As shown in Figure 6, the average accuracy rate of the martial arts body movement recognition method in this paper is 92.7%, and the average accuracy rates of the other two recognition methods are 80.4% and 82.9%, respectively.

In order to further reflect the performance of Wushu action recognition methods based on the features of bone points, the time-consuming statistics of the three methods are made, and the results are shown in the following table.

From the analysis of Table 2, it can be seen that the time consumed of the martial arts human body movement recognition method in this paper is 1.2 s and 1.41 s, respectively, which is much lower than the other two methods, indicating that the martial arts movement recognition method in this paper has higher recognition efficiency and better application performance.

## 4. Conclusion

In this paper, a recognition method of complex behaviors of Wushu human body based on bone point features is proposed. According to the multimodal classifier algorithm, the human body is divided into five parts, the variance of each part is calculated and sorted, and the bone points are determined according to the part with the largest variance. The feature of bone points is composed of different expressions of bone joints, which integrates various behavioral information such as kinetic energy, potential energy, joint direction, and joint angle, making the feature expression more effective. The experimental results show that the recognition accuracy of the research method for different types of movements is 90.1% and 92.7%, and the recognition time is 1.2 s and 1.41 s, which has superior recognition effect of Wushu movements. In this paper, the behavior recognition of large movements is effective, but the performance of subtle movement recognition is insufficient. In the follow-up, we can consider introducing the content of gesture recognition and fusing gestures with the features of limbs and torso to improve the recognition of subtle movements such as keyboard tapping.

## Figures and Tables

**Figure 1:** Wushu air leg movements.

**Figure 2:** Schematic diagram of the main generating muscles in the buffering phase.

**Figure 3:** Human movement recognition process.

**Figure 4:** Recognition effect diagram.

**Figure 5:** Recognition accuracy of msraction-3D data set (%).

**Figure 6:** Recognition accuracy of florence3D action data set (%).

**Table 1:** Node information of the 8 gateways.

1	Left shoulder	5	Left hip
	Left elbow		Left knee
2	Left shoulder	6	Left hip
	Left wrist		Left ankle
3	Right shoulder	7	Right hip
	Right elbow		Right knee
4	Right shoulder	8	Right hip
	Right wrist		Right ankle

**Table 2:** Time consumption of action recognition.

Method	msraction-3D data set	florence3D action data set
Recognition method of Wushu human complex movements based on neural network	8.54	9.73
Recognition method of Wushu human complex movements based on deep learning	10.36	12.37
The recognition method of complex movements of Wushu human body in this paper	1.2	1.41

## Data Availability

The data used and analyzed during the current study are available from the corresponding author on reasonable request.
